# Dose-response effect of prebiotic ingestion (β-glucans isolated from *Saccharomyces cerevisiae*) in diabetic rats with periodontal disease

**DOI:** 10.1186/s13098-021-00729-1

**Published:** 2021-10-18

**Authors:** Diana Vilela Azzi, Andressa Naira de Jesus Pereira, Viviam de Oliveira Silva, Renata de Carvalho Foureaux, Andressa Ribeiro Veiga Lima, Robson Sfaciotti Barducci, Adriana Silva Albuquerque, Gabriel Lasmar Reis, Raphael Ricon de Oliveira, Eric Francelino Andrade, Márcio Gilberto Zangeronimo, Antonio Chalfun-Júnior, Luciano José Pereira

**Affiliations:** 1 Department of Veterinary Medicine, Universidade Federal de Lavras (UFLA), Lavras, Minas Gerais Brazil; 2 Department of Research and Development, Biorigin Company, Macatuba, São Paulo Brazil; 3 Department of Biology, Universidade Federal de Lavras (UFLA), Lavras, Minas Gerais Brazil; 4 Institute of Agrarian Sciences, Universidade Federal dos Vales do Jequitinhonha e Mucuri (UFVJM), Unaí, Minas Gerais Brazil; 5 Department of Health Sciences, Universidade Federal de Lavras (UFLA), 3037, Lavras, Minas Gerais 37200-900 Brazil

**Keywords:** Periodontitis, Diabetes mellitus, Bone loss, Inflammatory status, β-glucans

## Abstract

**Background:**

Periodontal disease is one of the most frequent comorbidities in diabetic patients and can contribute to poor blood glucose control.

**Objective:**

To evaluate the effects of ingesting different doses of beta-glucans (BG) isolated from Saccharomyces cerevisiae on alveolar bone loss (ABL) and inflammatory/metabolic parameters in normal and diabetic rats with ligature-induced periodontal disease (PD).

**Design:**

Sixty male rats were assigned into two groups: non-diabetic or diabetic (i.p. 70 mg/kg streptozotocin) with PD. Then, groups were subdivided into five subgroups according BG doses: 0 mg/Kg; 10 mg/Kg; 20 mg/Kg; 40 mg/Kg or 80 mg/Kg. Animals received BG for 28 days and ligatures were placed on lower first molars during the last 14 days.

**Results:**

ABL of diabetic and non-diabetic animals receiving BG 40 mg/kg (1.33 ± 0.03 mm and 0.77 ± 0.07 mm, respectively) and 80 mg/kg (1.26 ± 0.07 mm and 0.78 ± 0.05 mm, respectively) doses was lower (p < 0.05) in comparison to respective controls (1.59 ± 0.11 mm and 0.90 mm ±0.08). COX-2 (Control: 1.66 ± 0.12; 40 mg/kg: 1.13 ± 0.07; 80 mg/kg: 0.92 ± 0.18) and RANKL expressions (Control: 1.74 ± 0.34; 40 mg/kg: 1.03 ± 0.29 ;80 mg/kg: 0.75 ± 0.21), together with the RANKL/OPG ratio (Control: 1.17 ± 0.08; 40 mg/kg: 0.67 ± 0.09; 80 mg/kg: 0.63 ± 0.28) were attenuated above the same dose (p < 0.05). BG did not influence (p > 0.05) metabolic parameters in non-diabetic rats. In diabetic animals, doses above 40 mg/kg reduced IL-1β (Control: 387 ± 66; 40 mg/kg: 309 ± 27; 80 mg/kg: 300 ± 14) and TNF-α (Control: 229 ± 19; 40 mg/kg: 128 ± 53; 80 mg/kg: 71 ± 25), blood glucose levels (Control: 402 ± 49; 40 mg/kg: 334 ± 32; 80 mg/kg: 287 ± 56), total cholesterol (Control: 124 ± 8; 40 mg/kg: 120 ± 10; 80 mg/kg: 108 ± 9), LDL-c + VLDL-c (Control: 106 ± 8; 40 mg/kg: 103 ± 10; 80 mg/kg: 87 ± 10) and triacylglycerols (Control: 508 ± 90; 40 mg/kg: 301 ± 40; 80 mg/kg: 208 ± 61), whereas increased HDL-c (Control: 18 ± 0.5; 40 mg/kg: 19 ± 1; 80 mg/kg: 21 ± 1) (p < 0.05). Optimal dose needed to reduce ABL was higher in diabetic animals with PD.

**Conclusions:**

BG ingestion reduced ABL and improved inflammatory profile in a dose-dependent manner. Best effects were achieved with doses above 40 mg/kg.

## Introduction

Periodontal disease (PD) is a group of inflammatory conditions initiated by the presence of disbiotic biofilm associated to teeth supporting tissues [1, 2]. Specific components of bacteria (e.g., lipopolysaccharide-LPS) stimulate periodontal cells to secrete several pro-inflammatory cytokines, including prostaglandins, IL-1, IL-6, TNF-α and endothelin [3], and promote bone loss through osteoclast activation. This process involves the expression of the receptor activator of nuclear factor kappa-Β ligand (*RANKL*) and reduced expression of osteoprotegerin (*OPG*) [4, 5].

Due to the common inflammatory pattern, evidence indicates a strong bidirectional relationship between PD and other chronic systemic diseases, such as diabetes mellitus (DM) [6]. Diabetic individuals are at higher risk and present more severe PD than healthy ones. As well, blood glucose control in diabetic patients is also hampered in the presence of PD [7]. Cytokines released in periodontal inflammation also influence insulin resistance and adipokines secretion [8]. In summary, PD and DM are two chronic non-transmissible diseases with significant impact on each other, impairing quality of life, reducing longevity and increasing health costs [9].

Alternative or supplementary treatments with functional foods such as probiotics and prebiotics have been studied to produce adjunctive periodontal benefits [10]. Prebiotics, such as beta-glucans (BGs), are non-digestible soluble fibers that are fermented by gut microbiota, producing short-chain fatty acids and inducing IgA secretion, enhancing the integrity of the intestinal barrier and host immunity [11]. BGs have demonstrated beneficial effects in preventing alveolar bone loss (ABL), with associated antidiabetic and other metabolic effects [8, 12, 13]. The main sources of BG’s are the cell walls of fungi, algae, bacteria, and cereals [14]. Depending on the source, they present different functional effects [13, 15]. Yeast-derived BGs have immunostimulant properties [16], by enhancing phagocytosis and modulating the production of inflammatory cytokines [14]. Previous studies from our group showed that daily doses (30 mg/kg/day for 28 days) of β-glucans from *Saccharomyces cerevisiae* reduced plasmatic levels of TNF-α [17] and ABL [8, 17] in animals with PD. In addition, BG reduced gingival expression of *Cyclooxygenase-2* and *RANKL* genes, whereas increased *OPG* expression in diabetic animals [8]. In animal models, doses employed for periodontal disease control varies from 10 mg/kg/day [18] to 85 mg/kg/day [19] in different studies. A dose-response effect and optimal dose are still unknown.

The Food and Drug Administration (FDA) considered yeast BG (isolated from *S.* *cerevisiae*) generally recognized as safe (GRAS) more than 10 years ago (Government Revenue Number: 000239). Maximum safe dose for consumption is 200 mg/per meal [20], ranging from 100 to 500 mg/day [15] Preclinical nutritional and toxicological studies play an indispensable role before proposing safe and efficacious startup dose for human studies [21]. Therefore, we aimed to evaluate the effects of different doses of BGs (*Saccharomyces cerevisiae*) on ABL, inflammatory and metabolic parameters of diabetic and nondiabetic rats with ligature-induced PD.

## Methods

### Animals

This study was approved by the Ethics Committee on Animal Use of the Federal University of Lavras, under Protocol 041/17. During experimental period, the animals were kept in polypropylene boxes (dimensions 41 cm × 34 cm × 17.5 cm), containing wood shavings, and maintained in acclimatized room (22 ± 2 °C; 45% ± 15% of humidity and 12–12 h light-dark cycle). Rodents received appropriate commercial feed and water ad libitum throughout the experimental period.

Sample size was determined based on ABL. The sample size was determined to provide 80% power to recognize a significant difference of 20% among groups and a standard deviation of 15% with a 95% confidence interval (α = 0.05) [8]. Therefore, a sample size of six animals per group was required. Sixty male Wistar rats (*Rattus norvegicus *albinus) with initial body weight ranging from 250 to 300 g were randomly assigned into two large groups: diabetic or non-diabetic. Diabetes was induced by intraperitoneal injection of streptozotocin (70 mg/kg). Each group (diabetic and non-diabetic) was subdivided into five subgroups of six animals/each according to the following BG doses: 0 mg/Kg; 10 mg/Kg; 20 mg/Kg; 40 mg/Kg or 80 mg/Kg.

### Administration of β-glucan

Animals received a commercial product containing BG isolated from *Saccharomyces cerevisiae* yeast by gavage, in accordance with respective experimental group, dissolved in 0.3 ml of filtered water for 28 consecutive days. Administration occurred always between 8 and 10 a.m. by the same researcher.

### Induction of experimental diabetes mellitus

DM induction was performed by intraperitoneal injection of 70 mg/kg of streptozotocin (Sigma, ST. Louis, MO, USA) dissolved in citrate buffer [22]. Forty-eight hours after induction, blood glucose was measured (8 h-fasting) through amputation of the tip of the tail using a glucometer (Accutrend^®^ Plus Roche, Basel, Switzerland). Animals with fasting blood glucose above 200 mg/dL [8] were considered diabetic. On the same day, BG administration started (Fig. 1).

**Fig. 1:** Schematic representation of the experimental model

### Periodontal disease induction

PD was induced using cotton thread ligatures around both right and left first mandibular molars. The animals were anesthetized using intraperitoneal injection of 10 mg/kg xylazine and 80 mg/kg ketamine [23]. Animals received BG for 28 days and PD was induced on the 15th day (Fig. 1).

### Euthanasia and collection of biological material

Euthanasia occurred by cardiac puncture after anesthesia (50 mg/kg of sodium thiopental i.p.). Blood was collected through cardiac puncture and the jaws were removed. The gingival tissue surrounding the first molars was immediately removed and stored at − 80 °C for gene expression analysis.

### Serum analyzes

Blood samples coagulated at room temperature. The tubes were centrifuged at RCF of 1252×*g* for 20 min. Serum was transferred into 2 ml tubes and stored in an ultra-freezer at − 80 °C until analysis. We determined blood glucose, total cholesterol (TC), triacylglycerols (TAG) and high-density lipoprotein cholesterol (HDL-C), using commercial enzymatic colorimetric kits (Labtest^®^, Lagoa Santa-MG, Brazil). LDL-C + VLDL-C levels of each animal were calculated using the following equation (CT– HDL = LDL + VLDL) [24]. Serum concentrations of TNF-α, IL-1β and IL-10 by immunoenzymatic assay (ELISA) were determined in diabetic animals using commercial kits (Invitrogen, Thermo-Fisher Inc., Vienna, Austria) and spectrophotometer (Epoch Biotek, Winooski, VT, USA).

### Morphometric analysis of alveolar bone resorption

The mandibles were collected to determine ABL using the morphometric method, after soft tissue removal [8] Initially, the pieces were fixed in 10% formalin solution. Subsequently, we immersed the samples in 30% hydrogen peroxide for 2 h to facilitate mechanical removal of the soft tissues. Staining was conducted using with 1% methylene blue for 1 min to delimit the cemento-enamel junction (CEJ).

The mandibles were observed in a stereomicroscope attached to a video camera and a computer. Images were stored with a 20× magnification. The distance between the alveolar bone crest and CEJ was measured in the central region of each root of the first molar from the lingual face following long axis [25] using the Image J software (Bethesda, MD, USA.). A trained examiner blind to all treatments made measurements. The average of the three measurements was used to express the degree of ABL for each animal.

### RT-qPCR analysis

Total RNA of gingival tissues surrounding the lower jaw first molars for non-diabetic animals was isolated using the Trizol^®^ reagent (Invitrogen, Life Technologies, USA). Subsequently, RNA quality and quantity were determined using a micro-volume spectrophotometer (Nanodrop 1000, Nanodrop technologies LLC, Wilmington, NC, USA). To assess the integrity of the samples, they were subjected to electrophoresis on 1.2% agarose gel stained with GelRed Nucleic Acid Gel Stain and visualized on a UV-transilluminator photo-documenter (UVITEC FireReader XS D-77Ls- 20. M). Reverse transcription of total DNA was used for cDNA synthesis with GoScript^TM^ Reverse Transcription kit (System Promega, Madison, WI, USA). Primer sets for the *COX2, RANKL, OPG* genes and for the *glyceraldehyde-3-phosphate dehydrogenase* (*GAPDH*) and *Beta actin* (*ACTB*) reference genes were designed from sequences available on GenBank using Primer Express 3.0 probe design software (Applied Bioystem, Foster City, CA, USA). Our reference genes were validated prior to use. Primers sequences were: *COX*-2: forward: 5′-CTCAGCCATGCAGCAAATCC-3′; reverse: 5′-GGGTGGGCTTCAGCAGTAAT-3′; *OPG*: forward: 5′-GGAATAGATGTCACCCTGTGCG-3′, reverse: 5′-AAGTTTGCTCTTGCGAGCTG-3′; *RANKL*: forward: 5′-ACATCCCATCGGGTTCCCATA-3′, reverse: 5′-AGCAAATGTTGGCGTACAGG-3′; *GAPDH*: forward: 5′-CCATCTTCCAGGAGCGAGA-3′, reverse: 5′-GGCGGAGATGATGACCCTTT-3′ and *ACTB*: forward: 5′-AGCCTTCCTTCCTGGGTATG-3′, reverse: 5′-CGGATGTCAACGTCACACTT-3′.

The quantification of the reaction product was performed using SYBR Green PCR Master Mix (Ferments, Glen Burnie, MD, USA) following the ddCT method and the averages were normalized in relation to the lowest value treatment for each gene. After quantifying the expression of *RANKL* and *OPG*, we calculated the RANKL/OPG ratio [26]. The RANKL/OPG ratio has been widely used as a parameter to quantify the severity of PD [26, 27].

### Statistical analysis

The data were submitted to the Anderson-Darling normality test, Breusch-Pagan homoscedasticity test and Durbin-Watson independence of errors test. Analysis of variance (ANOVA) were performed and when significant we conducted Dunnett test (at p < 0.05) in comparison to the control group (0 mg/Kg). We also compared ABL under different BG doses between non-diabetic and diabetic groups using two-way ANOVA. Regression analyses were conducted determine the optimal dose able to prevent ABL in non-diabetic and diabetic animals. We used Action software (Estatcamp, version 3.4, São Carlos, São Paulo, Brazil).

## Results

ABL of diabetic and non-diabetic animals receiving BG 40 mg/kg (1.33 ± 0.03 mm and 0.77 ± 0.07 mm, respectively) and 80 mg/kg (1.26 ± 0.07 mm and 0.78 ± 0.05 mm, respectively) doses was lower (p < 0.05) in comparison to respective controls (1.59 ± 0.11 mm and 0.90 mm ±0.08) (Fig. 2A–L). The ideal dose of BG ingestion was 54 mg/Kg for non-diabetic animals (Fig. 2A), whereas the best dose for diabetic was 80 mg/kg (Fig. 2G). ABL was higher in diabetic animals with PD (compared to non-diabetic animals) for all tested doses. Two-way ANOVA indicated significant interaction between diabetes and BG dose (p < 0.05; Fig. 3).

**Fig. 2:** Regression analyses of alveolar bone resorption in non-diabetic (**A**) and diabetic rats with ligament-induced periodontal disease (**G**) and treated with different doses of *Saccharomyces cerevisiae* β-glucan for 28 days, respectively. **B**–**F** Representation of alveolar bone resorption in non-diabetic animals with ligature-induced periodontal disease and treated with different levels of *Saccharomyces cerevisiae* β-glucan for 28 days. **B** control (0 mg/kg). JCE (Enamel cement junction), COA (Alveolar bone crest). **C** (10 mg/Kg). **D** (20 mg/Kg). **E** (40 mg/Kg). **F** (80 mg/Kg). **H–L** Representation of alveolar bone resorption in diabetic animals with ligature-induced periodontal disease and treated with different levels of *Saccharomyces cerevisiae* β-glucan for 28 days. **H** diabetic (0 mg/kg). **I** (10 mg/Kg). **D** (20 mg/Kg). **E** (40 mg/Kg). **F** (80 mg/Kg)

**Fig. 3:** Two-way ANOVA comparing alveolar bone loss between diabetic and non-diabetic animals treated with different doses of *Saccharomyces cerevisiae* β-glucan for 28 days. *Differs from control group (0 mg/Kg) by Dunnett test (p < 0.05). ^#^Differs from non-diabetic groups. ^§^Significant effect of doses

The *RANKL* expression (Control: 1.74 ± 0.34; 40 mg/kg: 1.03 ± 0.29 ;80 mg/kg: 0.75 ± 0.21) and RANKL/OPG ratio (Control: 1.17 ± 0.08; 40 mg/kg: 0.67 ± 0.09; 80 mg/kg: 0.63 ± 0.28) in non-diabetic rats decreased (p < 0.05) at 40 and 80 mg/kg in comparison to animals not receiving BG (Fig. 4A, D). *OPG* expression was not altered (p > 0.05) by BG ingestion (Fig. 4B). The gingival expression of *COX-2* (Control: 1.66 ± 0.12; 40 mg/kg: 1.13 ± 0.07; 80 mg/kg: 0.92 ± 0.18) was attenuated (p <0.05) from 20 mg/kg doses (Fig. 4C).

**Fig. 4:** Relative expression of **A** *RANKL*, **B** *OPG*, **C** *COX-2*, and **D** RANKL/OPG ratio in rats with ligature-induced periodontal disease and treated with different doses of *Saccharomyces cerevisiae* β-glucan for 28 days. *Differs from control group (0 mg/Kg) by Dunnett test (p < 0.05)

Metabolic variables such as TAG, CT, HDL-c and LDL-C + VLDL-c remained unchanged among non-diabetic groups, independently of BG dose ingestion (Fig. 5A–D). However, for diabetic animals, 40 mg/kg and 80 mg/kg reduced (p < 0.05) blood glucose (Control: 402 ± 49; 40 mg/kg: 334 ± 32; 80 mg/kg: 287 ± 56) and TAG levels (Control: 508 ± 90; 40 mg/kg: 301 ± 40; 80 mg/kg: 208 ± 61) (Fig. 6A, E). HDL-C levels increased (Control: 18 ± 0.5; 40 mg/kg: 19 ± 1; 80 mg/kg: 21 ± 1) (p < 0.05) while TC (Control: 124 ± 8; 40 mg/kg: 120 ± 10; 80 mg/kg: 108 ± 9) and LDL-C + VLDL-C levels (Control: 106 ± 8; 40 mg/kg: 103 ± 10; 80 mg/kg: 87 ± 10) decreased (p < 0.05) for animals receiving 80 mg/kg (Fig. 6C, B, D).

**Fig. 5:** Biochemical parameters of non-diabetic rats with ligature-induced periodontal disease and treated with different doses of *Saccharomyces cerevisiae* β-glucan for 28 days. **A** Total cholesterol. **B** HDL-c. **C** LDL-c +VLDL-c. **D** Triacylglycerol

**Fig. 6:** Biochemical parameters of diabetic (STZ) rats with ligature-induced periodontal disease and treated with different doses of *Saccharomyces cerevisiae* β-glucan for 28 days. **A** Blood glucose. **B** Total cholesterol. **C** HDL-c. **D** LDL-c +VLDL-c. **E** Triacylglycerol. *Differs from control group (0 mg/Kg) by Dunnett test (p < 0.05)

Serum levels of IL-1β (Control: 387 ± 66; 40 mg/kg: 309 ± 27; 80 mg/kg: 300 ± 14) and TNF-α (Control: 229 ± 19; 40 mg/kg: 128 ± 53; 80 mg/kg: 71 ± 25) decreased (p < 0.05) with 40 mg/kg and 80 mg/kg ingestion in diabetic groups (Fig. 7A, B). IL-10 (Fig. 7C) levels increased (p < 0.05) and IL-1β/IL-10 and TNF-α/IL-10 ratios decreased (p < 0.05) from the smallest tested dose of 10 mg/kg (Fig. 7D, E).

**Fig. 7:** Immunological parameters of diabetic (STZ) rats with ligature-induced periodontal disease and treated with different doses of *Saccharomyces cerevisiae* β-glucan for 28 days. **A** IL-1β. **B** TNF-α. **C** IL-10. **D** IL-1β/IL-10 ratio. **E** TNF-α/ IL-10 ratio. *Significantly differs from the control group (0 mg/Kg) by the Dunnett test (p < 0.05)

## Discussion

This study demonstrated for the first time that BG effects on ABL is dose-dependent. Additionally, we observed that diabetic animals with PD needed higher doses than non-diabetic ones. Indeed, DM worsens ABL, confirming the bidirectional relationship between the two diseases.

ABL is attributed to an inflammatory host response against biofilm dysbiosis [28]. BG doses of 40 mg/kg or greater were the most effective in attenuating ABL in both non-diabetic and diabetic rats. This result was associated to a reduction in the expression of *COX-2*, *RANKL* and RANKL/OPG ratio. Such outcomes reinforced the idea that BG can modulate the gingival inflammatory profile and mitigate ABL ligature-induced periodontitis [8, 17, 19].

RANKL interacts with its receptor on the surface of osteoclast precursor cells (monocytes) leading to its differentiation and stimulating its resorptive activity [29]. In parallel, a reduction in the expression of *OPG* by osteoblasts, increases the differentiation and activation of osteoclasts [30]. A higher expression of *RANKL* and an elevated RANKL/OPG ratio indicate greater inflammation and greater bone loss, whereas the contrary indicates a protective effect for alveolar bone.[26] We observed that the administration of BG at the highest doses (40 and 80 mg/kg) attenuated *RANKL* expression. This behavior reflected in the reduction of RANKL/OPG ratio, indicating the protective properties of BG against ABL [31].

ABL attenuation associated to increased BG ingestion was also consistent with reduced *COX-2* gene expression. *COX-2* in the gums has been linked to prostaglandins (especially PGE2) production and to a worse PD prognosis [32] Prostaglandins produced by osteoblasts and other cells of the periodontal ligament are potent stimulators of bone resorption [32] and epithelial insertion losses in periodontal disease [33].

The expression of *COX-2*, *RANKL* and *OPG* can be regulated by local and systemic stimuli, through hormones, inflammatory mediators, drugs and substances produced by bacteria, and are considered important molecular targets for therapeutic intervention [27, 30]. In our study, the ideal BG dose observed for ABL control in non-diabetic rats was 54 mg/kg. The literature shows for various metabolic and immune conditions, variations in BG doses from 0.1 to 20 mg/kg for humans and from 10 to 1250 mg/kg in an animal model [34]. However, few studies have investigated the effects of different doses of BG on ligature-induced periodontitis. As example, Kim et al. [19] evaluated oral 21.25; 42.5 and 85 mg/kg doses of Polycan (a purified BG from *Aureobasidium pullulans*), with effective results in preventing ABL only for the two higher doses. However, a regression model or optimal dose was not determined.

As diabetes involves systemic bidirectional relationship with PD, we evaluated plasmatic inflammatory mediators in those animals and their influence on ABL and metabolic parameters. Doses above 40 mg/kg were the most effective in reducing ABL and serum levels of IL-1β and TNF-α. The inflammatory response of PD involves high levels of pro-inflammatory cytokines such as IL-1β and TNF-α [35]. IL-1β participates in the activation of endothelial cells allowing the adhesion of eosinophils, increasing the inflammatory response and regulating the production and activity of osteoclasts. IL-1β levels are higher in individuals with periodontitis [36]. In addition, elevated levels of TNF-α stimulate osteoclastogenesis, increasing the production of macrophage colony stimulating factor (MCS-F) and RANKL in bone marrow stromal cells, osteoblasts and lymphocytes [37]. TNF-α increases RANKL/OPG ratio favoring bone loss [38]. High IL-1β/IL-10 and TNF-α/IL-10 ratios are associated with greater bone resorption in PD [39]. Our results from diabetic animals showed increased serum concentrations of the anti-inflammatory cytokine (IL-10), with a consequent reduction in the IL-1β/IL-10 and TNF-α/IL-10 ratios starting from the smallest 10 mg/kg dose. IL-10 plays a key role in suppressing TNF-α and IL-1β, acting as a tissue inhibitor of metalloproteinases and prostaglandin E, in addition to promoting the expression of anti-inflammatory receptor mediators as the interleukin 1 receptor antagonist.

This immunomodulatory effect of BGs seems to be attributed to its fermentation by the intestinal microbiota and the production of short-chain fatty acids (SCFA), generating a systemic anti-inflammatory effect [35]. SCFA in the intestinal lumen can cross the epithelium by diffusion and interact with surface molecules in the immune cells of the lamina propria or bind to protein G receptors (GRP41 and GRP43) coordinating various signaling and regulatory pathways of gene expression associated gut-associated lymphoid tissue (GALT) [40]. SCFA may modulate T cell activity in inflammatory conditions [41]. by inhibiting histone deacetylases (HDACs), as well as acting as substrates for generation of acetyl Coa, which are essential mechanisms for cytokine gene expression [42]. In short, the generation of SCFA promotes a reduction in IL-1β and TNF-α and increased secretion of IL-10, reducing the activation of nuclear factor kappa-B (NF-kB) [43] and consequently decreasing the systemic inflammatory response, which is of great importance in chronic inflammatory diseases [40].

BG ingestion did not promote significant changes in the metabolic parameters evaluated in non-diabetic animals (CT, TAG, HDL-c and LDL-c + VLDL-c). This result is similar to that observed in previous studies in healthy animals [13, 23] and humans [44, 45]. Results from our group demonstrated negative effects of PD on metabolic parameters of rats, such as reduction in pancreatic beta cell function and increased serum levels of TNF-α even in non-diabetic rats [17]. These alterations were still within the normal reference levels during the 14 days of PD induction [46] or dyslipidemia [24]. However, when PD was induced in diabetic animals, metabolic disruption worsened [17].

In the present study we observed in diabetic animals that the highest dose (80 mg/kg) of BG promoted the best benefits for blood concentrations of TAG, LDL-c + VLDL-c, TC and HDL-c. BGs reduces LDL-c by blocking the micelles of bile acids, impairing their ability to interact with luminal membrane transporters in the intestinal epithelium and decreasing their absorption with a consequent increase in fecal cholesterol [47]. Subsequently, the reduction of bile acids causes an increase in the expression of the enzyme cholesterol 7α-hydroxylase in the liver, which positively regulates the low-density lipoprotein receptor (LDL-R). In this way, the transport of LDL-c in hepatocytes increases and so the conversion of cholesterol into bile acids further contributing to LDL-c reduction [48]. Our results also showed a significant decrease in blood glucose in the 40 mg/kg dose of BG in diabetic rats, probably due to the formation of a gelatinous layer in the intestine, reducing carbohydrates and lipids absorption [49]. The larger the layer is, the lower the glucose uptake will be, and this fact explains why larger doses have better anti-diabetic effects [14]. In addition, BGs promote suppression of the glucose and sodium transporter (SGLT-1) in the intestinal mucosa; modulate the intestinal microbiota; reduce the activity of intestinal disaccharidases (especially at higher doses of BG) [50], improving the activity of the enzyme Succinate dehydrogenase. All these mechanisms contribute to reducing blood glucose levels [50].

Although there are several studies on the metabolic and immunomodulatory effects of BGs [8, 12, 13] none has investigated the optimal dose for DM and PD comorbidities. Several doses are reported in the literature [8, 13, 34]. No toxic or adverse effects were observed after subchronic administration of BG doses up to 100 mg/kg [34]. In addition, in animal models, oral administration of BGs has been used to decrease toxicity of mercury, methotrexate and paracetamol [34]. Although we evaluated doses starting at 10 mg/kg, those above 40 mg/kg were the most effective in reducing PD and controlling systemic metabolic/inflammatory diseases. Our results suggest that effective BGs doses are influenced by pre-existing health condition and that diabetic individuals may need greater BG doses to achieve better results.

## Conclusions

Treatment with BGs attenuates ABL and improves local and systemic inflammatory parameters at doses above 40 mg/kg. Diabetic animals needed higher BG doses to achieve the same results as normal animals.

## Data Availability

The datasets used and/or analysed during the current study are available from the corresponding author on reasonable request.

## References

[1] AAP. American Academy of Periodontology Task (2015). Force report on the update to the 1999 classification of periodontal diseases and conditions. J Periodontol.

[2] Park SI, Kang SJ, Han CH, Kim JW, Song CH, Lee SN (2016). The effects of topical application of Polycal (a 2:98 (g/g) mixture of Polycan and calcium gluconate) on experimental periodontitis and alveolar bone loss in rats. Molecules.

[3] Breivik T, Thrane PS, Murison R, Gjermo P (1996). Emotional stress effects on immunity, gingivitis and periodontitis. Eur J Oral Sci.

[4] Crotti TN, Dharmapatni AASSK, Alias E, Haynes DR (2015). Osteoimmunology: major and costimulatory pathway expression associated with chronic inflammatory induced bone loss. J Immunol Res.

[5] Savage A, Eaton KA, Moles DR, Needleman I (2009). A systematic review of definitions of periodontitis and methods that have been used to identify this disease. J Clin Periodontol.

[6] Gaudilliere DK, Culos A, Djebali K, Tsai AS, Ganio EA, Choi WM (2019). Systemic immunologic consequences of chronic periodontitis. J Dent Sci.

[7] Liccardo D, Cannavo A, Spagnuolo G, Ferrara N, Cittadini A (2019). Periodontal disease: a risk factor for diabetes and cardiovascular disease. Int J Mol Sci.

[8] Silva VO, Lobato RV, Andrade EF, De Macedo CG, Napimoga JTC, Napimoga MH (2015). β-Glucans (*Saccharomyces cereviseae*) reduce glucose levels and attenuate alveolar bone loss in diabetic rats with periodontal disease. PLoS ONE.

[9] Quintero AJ, Sanz A, Chaparro A, Quirynen M, Ramirez V, Prieto D (2018). Effect of two periodontal treatment modalities in patients with uncontrolled type 2 diabetes mellitus: a randomized clinical trial. J Clin Periodontol.

[10] Foureaux R, de Messora C, de Oliveira MR, Napimoga LFF, Pereira MH, Ferreira ANJ (2014). Effects of probiotic therapy on metabolic and inflammatory parameters of rats with ligature-induced periodontitis associated with restraint stress. J Periodontol.

[11] Davani-Davari D, Negahdaripour M, Karimzadeh I, Seifan M, Mohkam M, Masoumi SJ (2019). Prebiotics: definition, types, sources, mechanisms, and clinical applications. Foods.

[12] Silva VO, Moura NO, Oliveira LJR, Peconick AP, Pereira LJ (2017). Promissing effects of beta-glucans on metabolism and on the immune responses: review article. Am J Immunol.

[13] Vieira Lobato R, De Oliveira Silva V, Francelino Andrade E, Ribeiro Orlando D, Gilberto Zangeronimo M, Vicente de Sousa R (2015). Metabolic effects of β-glucans (*Saccharomyces cerevisae*) per os administration in rats with streptozotocin-induced diabetes. Nutr Hosp.

[14] Francelino Andrade E, Vieira Lobato R, Vasques Araújo T, Gilberto Zangerônimo M, Vicente Sousa R, José Pereira L (2014). Effect of beta-glucans in the control of blood glucose levels of diabetic patients: a systematic review. Nutr Hosp.

[15] Vetvicka V, Vannucci L, Sima P, Richter J (2019). Beta glucan: supplement or drug? From laboratory to clinical trials. Molecules.

[16] Miura NN, Adachi Y, Yadomae T, Tamura H, Tanaka S, Ohno N (2003). Structure and biological activities of β-glucans from yeast and mycelial forms of *Candida albicans*. Microbiol Immunol.

[17] Silva VO, Lobato RV, Andrade EF, Orlando DR, Borges BDB, Zangeronimo MG (2017). Effects of β-glucans ingestion on alveolar bone loss, intestinal morphology, systemic inflammatory profile, and pancreatic β-cell function in rats with periodontitis and diabetes. Nutrients.

[18] Breivik T, Opstad PK, Engstad R, Gundersen G, Gjermo P, Preus H (2005). Soluble β-1,3/1,6-glucan from yeast inhibits experimental periodontal disease in Wistar rats. J Clin Periodontol.

[19] Kim YS, Kang SJ, Kim JW, Cho HR, Moon SB, Kim KY (2012). Effects of Polycan, a β-glucan, on experimental periodontitis and alveolar bone loss in Sprague-Dawley rats. J Periodontal Res.

[20] Thompson IJ, Oyston PCF, Williamson DE (2010). Potential of the β-glucans to enhance innate resistance to biological agents. Expert Rev Anti Infect Ther.

[21] Guha R (2016). Preclinical pharmacology and toxicology: an important aspect in drug discovery. Adv Clin Toxicol.

[22] Hendarto H, Inoguchi T, Maeda Y, Ikeda N, Zheng J, Takei R (2012). GLP-1 analog liraglutide protects against oxidative stress and albuminuria in streptozotocin-induced diabetic rats via protein kinase A-mediated inhibition of renal NAD(P)H oxidases. Metabolism.

[23] Messora MR, Oliveira LFF, Foureaux RC, Taba M, Zangerônimo MG, Furlaneto FAC (2013). Probiotic therapy reduces periodontal tissue destruction and improves the intestinal morphology in rats with ligature-induced periodontitis. J Periodontol.

[24] de Araújo TV, Andrade EF, Lobato RV, Orlando DR, Gomes NF, de Sousa RV (2017). Effects of beta-glucans ingestion (*Saccharomyces cerevisiae*) on metabolism of rats receiving high-fat diet. J Anim Physiol Anim Nutr.

[25] Crawford JM, Taubman MA, Smith DJ (1978). The natural history of periodontal bone loss in germfree and gnotobiotic rats infected with periodontopathic microorganisms. J Periodontal Res.

[26] Cochran DL (2008). Inflammation and bone loss in periodontal disease. J Periodontol.

[27] Bostanci N, İlgenli T, Emingil G, Afacan B, Han B, Töz H (2007). Gingival crevicular fluid levels of RANKL and OPG in periodontal diseases: implications of their relative ratio. J Clin Periodontol.

[28] Taubman MA, Valverde P, Han X, Kawai T (2005). Immune response: the key to bone resorption in periodontal disease. J Periodontol.

[29] Liu D, Xu JK, Figliomeni L, Huang L, Pavlos NJ, Rogers M (2003). Expression of RANKL and OPG mRNA in periodontal disease: possible involvement in bone destruction. Int J Mol Med.

[30] Gibertoni F, Sommer MEL, Esquisatto MAM, do Amaral MEC, de Oliveira CA, de Andrade TAM (2017). Evolution of periodontal disease: immune response and RANK/RANKL/OPG system. Braz Dent J.

[31] Crotti T, Smith MD, Hirsch R, Soukoulis S, Weedon H, Capone M (2003). Receptor activator NF κB ligand (RANKL) and osteoprotegerin (OPG) protein expression in periodontitis. J Periodontal Res.

[32] Kayal RA (2013). The role of osteoimmunology in periodontal disease. Biomed Res Int.

[33] Tsai YL, Chang MC, Lin LD, Chan CP, Wang CY, Lin PS (2014). Stimulation of prostanoids and IL-8 production in human gingival fibroblasts by *Porphyromonas gingivalis* LPS is associated with MEK/ERK signaling. J Dent Sci.

[34] Samuelsen ABC, Schrezenmeir J, Knutsen SH (2014). Effects of orally administered yeast-derived beta-glucans: a review. Mol Nutr Food Res.

[35] Ratajczak W, Rył A, Mizerski A, Walczakiewicz K, Sipak O, Laszczyńska M (2019). Immunomodulatory potential of gut microbiome-derived short-chain fatty acids (SCFAs). Acta Biochim Pol.

[36] Aral K, Milward MR, Cooper PR (2020). Inflammasomes and their regulation in periodontal disease: a review. J Periodontal Res.

[37] Marahleh A, Kitaura H, Ohori F, Kishikawa A, Ogawa S (2019). TNF-α directly enhances osteocyte RANKL expression and promotes osteoclast formation. Front Immunol.

[38] Boyce BF, Xing L (2009). Functions of RANKL/RANK/OPG in bone modeling and remodeling. Arch Biochem Biophys.

[39] Passoja A, Puijola I, Knuuttila M, Niemelä O, Karttunen R, Raunio T (2010). Serum levels of interleukin-10 and tumour necrosis factor-α in chronic periodontitis. J Clin Periodontol.

[40] Koh A, De Vadder F, Kovatcheva-Datchary P, Bäckhed F (2016). From dietary fiber to host physiology: short-chain fatty acids as key bacterial metabolites. Cell.

[41] Haghikia A, Jörg S, Duscha A, Berg J, Manzel A, Waschbisch A (2015). Dietary fatty acids directly impact central nervous system autoimmunity via the small intestine. Immunity.

[42] Tanoue T, Atarashi K, Honda K (2016). Development and maintenance of intestinal regulatory T cells. Nat Rev Immunol.

[43] Browne HP, Neville BA, Forster SC, Lawley TD (2018). Europe PMC Funders Group Transmission of the gut microbiota: spreading of health. Nat Rev Microbiol.

[44] Chen J, He J, Wildman RP, Reynolds K, Streiffer RH, Whelton PK (2006). A randomized controlled trial of dietary fiber intake on serum lipids. Eur J Clin Nutr.

[45] Frank J, Sundberg B, Kamal-Eldin A, Vessby B, Aman P (2004). Yeast-leavened oat breads with high or low molecular weight beta-glucan do not differ in their effects on blood concentrations of lipids, insulin, or glucose in humans. J Nutr.

[46] Andrade EF, Orlando DR, Gomes JAS, Foureaux R, de Costa C, Varaschin RC (2017). Exercise attenuates alveolar bone loss and anxiety-like behaviour in rats with periodontitis. J Clin Periodontol.

[47] Tosun D, Siddarth P, Toga AW, Hermann B, Caplan R (2011). Effects of childhood absence epilepsy on associations between regional cortical morphometry and aging and cognitive abilities. Hum Brain Mapp.

[48] Cicero AFG, Fogacci F, Veronesi M, Strocchi E, Grandi E, Rizzoli E (2020). A randomized placebo-controlled clinical trial to evaluate the medium‐term effects of oat fibers on human health: the beta‐glucan effects on lipid profile, glycemia and intestinal health (BELT) study. Nutrients.

[49] Reyna NY, Cano C, Bermúdez VJ, Medina MT, Souki AJ, Ambard M (2003). Sweeteners and beta-glucans improve metabolic and anthropometrics variables in well controlled type 2 diabetic patients. Am J Ther.

[50] Jilin Dong F, Ruiling Shen CYL (2011). Hypoglycaemic effects and inhibitory effect on intestinal disaccharidases of oat beta-glucan in streptozotocin-induced diabetic mice. Food Chem.

